The article "Efficacy of Jiedu Pingsou Decoction Combined with Azithromycin in the Treatment of Children with Mycoplasma Pneumonia and Its Effects on Inflammatory Factors and Immune Function" was retracted in 2023. Reasons: unreliable results or conclusions; concerns about the data; concerns about the peer review; concerns about the citations.

# Efficacy of Jiedu Pingsou Decoction Combined with Azithromycin in the Treatment of Children with Mycoplasma Pneumonia and Its Effects on Inflammatory Factors and Immune Function

**DOI:** 10.1155/2022/9102727

**Published:** 2022-03-24

**Authors:** Shaoli Lin, Shiyun Wang, Juan Zhang, Min Zhuang, Zhen Meng, Jianhua Liu

**Affiliations:** ^1^Department of Pediatrics, Yantaishan Hospital, Yantai 264000, Shandong, China; ^2^Department of Pediatrics (I), Jiyang People's Hospital, Jinan 251400, Shandong, China; ^3^Department of Traditional Chinese Medicine, Qingdao Eighth People's Hospital, Qingdao 266000, Shandong, China; ^4^Department of Endocrinology, Zhangqiu District People's Hospital, Jinan 250200, Shandong, China; ^5^Department of Ultrasound, Zhangqiu District People's Hospital, Jinan 250200, Shandong, China; ^6^Infirmary of Veteran Cadre Rest Center, Zhangqiu District People's Hospital, Jinan 250200, Shandong, China

## Abstract

**Objective:**

The purpose of this study is to detect the clinical efficacy of Jiedu Pingsou Decoction combined with azithromycin in the treatment of children with mycoplasma pneumonia and the effect on inflammatory factors and immune function in children.

**Methods:**

A total of 68 children with mycoplasma pneumonia in our hospital from January 2021 to January 2022 were included in this study, and they were randomly divided into the control group and the observation group with 34 cases in each group. The children in the control group were treated with azithromycin, and the children in the observation group were treated with Jiedu Pingsou Decoction on this basis. The clinical manifestations, treatment effects, blood routine, serum inflammatory factor levels, and T cell subsets before and after treatment were compared between the two groups.

**Results:**

The total effective rate in the observation group was 94.12%, which was higher than that in the control group, which was 82.35%, and the difference between the two groups was statistically significant (*P* < 0.05). After treatment, the levels of CD3+, CD4+, and CD4+/CD8+ in the two groups were higher than those before treatment, and the level of CD8+ was lower than before treatment. The difference between groups was statistically significant (*P* < 0.05). The levels of serum C-reactive protein (CRP), tumor necrosis factor-*α* (TNF-*α*), interferon gamma (IFN-*γ*), interleukin-6 (IL-6), and interleukin-10 (IL-10) in the two groups after treatment were lower than those before treatment, and the difference between the two groups was statistically significant (*P* < 0.05). The difference between groups was statistically significant (*P* < 0.05). There were 4 cases and 2 cases of adverse reactions in the control group and the observation group, respectively, and the difference between the two groups was statistically significant (*P* > 0.05).

**Conclusion:**

Jiedu Pingsou Decoction combined with azithromycin can effectively improve the levels of T cell subsets, immune function, and inflammatory factors in children with mycoplasma pneumonia, improve clinical symptoms, and is safe and stable, and can be used in clinical practice.

## 1. Introduction

*Mycoplasma pneumoniae* (MP) is an important pathogen of respiratory tract infections in childhood [1, 2]. The main routes of transmission of *Mycoplasma pneumoniae* are respiratory droplets and aerosols. Children infected with *Mycoplasma pneumoniae* experience upper respiratory tract infections, rhinitis, pharyngitis, bronchitis, and pneumonia. Long-term unhealing can easily lead to complications such as atelectasis and pleural effusion, which not only seriously affects the respiratory function of children [3] but also affects other system functions of the body, and the life and health of children are greatly threatened. The epidemic season of *Mycoplasma pneumoniae* has certain regional and territorial characteristics [4, 5]. It is known that the global infection rate is as high as 60% or more, and there is a trend of increasing year by year [6–8].

Western medicine treatment of *Mycoplasma pneumoniae* is mainly based on macrolides, and the commonly used drug is azithromycin. However, long-term use of azithromycin can cause discomfort to the gastrointestinal tract in children, and it is prone to drug resistance. Combined with mixed infection, mycoplasma colonization, and many other factors, the Western medicine treatment of mycoplasma pneumonia has caused great difficulties and affected the therapeutic effect [9–12]. With the deepening of clinical understanding of traditional Chinese medicine, more and more studies have used it in the treatment of children with mycoplasma pneumonia [13]. The role of traditional Chinese medicine in suppressing inflammation, enhancing immunity, and relieving cough has been gradually recognized. In the treatment of diseases, Chinese medicine, starting from the overall concept, advocates treatment based on syndrome differentiation and the principle of seeking the basis of treatment, shortening the course of treatment, and speeding up the recovery process of the body. Traditional Chinese medicine can reduce the recurrence rate and improve the long-term prognosis of children by consolidating the root.

This article explores 68 children with mycoplasma pneumonia diagnosed and treated in our hospital from January 2021 to January 2022. The purpose of this study is to further explore and analyze the effects of Jiedu Pingsou Decoction combined with azithromycin on inflammatory factors and immune function on the basis of previous research and to evaluate its corresponding clinical efficacy.

## 2. Materials and Methods

### 2.1. Study Subjects and Groupings

All the children were outpatient or inpatient in our hospital from January 2021 to January 2022, with a total of 68 cases, and were divided into the control group and the observation group with 34 cases in each group according to the random number table method. The control group consisted of 21 males and 13 females, aged 3–11 (7.32 ± 2.13) years, and the disease duration was 2–9 (6.26 ± 1.21) days. The observation group included 20 males and 14 females, aged 3–11 (7.29 ± 2.10) years old, and the course of disease was 4–9 (6.24 ± 1.23) days. There was no significant difference in general data between the two groups (*P* > 0.05), and they were comparable, as shown in Table 1. All the specimens of this study were got the informed consent from patients and were approved by the Ethical Committee of our hospital.

### 2.2. Diagnostic Criteria

(1) The diagnostic standard of Western medicine is based on the standard of “Zhu Futang Practical Pediatrics.” (2) The traditional Chinese medicine (TCM) diagnostic criteria are based on the “Interpretation of TCM Clinical Treatment Guidelines (Paediatric Diseases)” standard.

### 2.3. Inclusion Criteria

Children who meet the diagnostic criteria for mycoplasma pneumonia and are confirmed by bacterial culture experiments were included. The children were 2–14 years old, and the families of the enrolled children gave informed consent to this study.

### 2.4. Exclusion Criteria

Children with respiratory tract infection not caused by *Mycoplasma*; children with pulmonary tuberculosis; children with severe heart, brain, and kidney diseases; children with respiratory failure; and children allergic to the drugs in this study were excluded.

### 2.5. Treatment

The children in the control group were routinely given azithromycin intravenously or orally for 2 weeks. The children in the observation group were treated with Chinese medicine Jiedu Pingsou Decoction on this basis. Prescription drugs: choose gypsum 5–20 g, trichosanthin 3–5 g, skullcap 3–5 g, platycodon 3–5 g, houttuynia cordata 3–6 g, honeysuckle 3–6 g, golden buckwheat root 5–10 g, 3–5 g of *Fritillaria fritillary*, 3–10 g of melon, 3–5 g of dried tangerine peel, 3–5 g of citrus aurantium, 3–10 g of northern ginseng, 6 g of almond, 3–6 g of ginger, and 2–3 g of licorice. The clinical evidence can be adjusted according to the specific condition of the child. The above prescription is taken 1 dose daily for 2 weeks.

### 2.6. Observation Indicators

#### 2.6.1. Inflammatory Factors

Blood routine related indicators (WBC), before and after treatment, and the patient's white blood cell (WBC), hemoglobin (Hb), and platelet (PLT) counts were detected. The levels of inflammatory factors were measured by double-antibody sandwich ELISA. The inflammatory factors were C-reactive protein (CRP), tumor necrosis factor-*α* (TNF-*α*), interferon-*γ* (INF-*γ*), interleukin-6 (IL-6), and interleukin-10 (IL-10).

#### 2.6.2. Changes in T Lymphocyte Subset-Related Indicators (CD3+, CD4+, CD8+, and CD4+/CD8+)

Before and after treatment, 5 mL fasting venous blood was collected and placed on an automatic blood centrifuge for centrifugation. The speed of the centrifuge was adjusted to 3000 r/min for 10 min, and the supernatant was taken and placed in a −20°C refrigerator for testing. Flow cytometry was utilized to measure T lymphocyte subsets-related indicators in serum.

### 2.7. Efficacy Criteria

The evaluation was based on the curative effect standard of “pneumonia asthma” in “Traditional Chinese Medicine Disease Syndrome Diagnosis and Efficacy Standards” formulated by the State Administration of Traditional Chinese Medicine. Significant effective: the chest X-ray examination showed that the child returned to normal, the body temperature and blood routine returned to normal, and the relevant clinical symptoms and signs disappeared. Effective: the chest X-ray examination of the child showed that the lung shadow was reduced but still visible, and the blood routine examination still showed signs of infection, and the related clinical symptoms and signs were relieved. Ineffective: the chest X-ray examination showed increased shadows in the lungs, and related clinical symptoms and signs were not relieved or even aggravated. Total effective rate = (marked number + effective number)/total number of cases × 100%

### 2.8. TCM Symptom Score

Before and after treatment, referring to “Chinese Medicine Emergencies,” it is divided into main syndrome scores: cough, body temperature, sputum, and tongue coating. The scoring standard is calculated from 0 to 6 points for each sign and symptom, and 2 points are added for each symptom aggravation. Secondary syndrome scores: vomiting, abdominal pain, thirst, sleep, and spirit. The scoring standard is based on the above symptoms ranging from 0 to 3 points, and each time the symptoms are aggravated on the basis of the original symptoms, 1 point will be added.

### 2.9. Incidence of Adverse Reactions

The incidence of vomiting and diarrhea in the two groups after treatment were compared.

### 2.10. Statistical Methods

Measurement data were expressed as mean ± standard deviation. Enumeration data were expressed in the form of cases or percentages, and the *χ*^2^ test was used. Data analysis was processed with SPSS 22.0 statistical analysis software. The *t*-test was used to test the data between the same groups. *P* < 0.05 means the difference is statistically significant.

## 3. Results

### 3.1. Comparison of the Clinical Efficacy of the Two Groups of Patients

The clinical symptoms of the two groups were relieved after treatment, the effective rate of the control group was 82.35%, and the effective rate of the observation group was 94.12%. The effective rate of the two groups was compared, and the difference was statistically significant (*P* < 0.05), as shown in Table 2.

### 3.2. Comparison of Clinical Symptom Scores between the Two Groups before and after Treatment

There was no significant difference in clinical symptom scores before treatment between the two groups (*P* > 0.05). After treatment, the clinical symptom scores of the observation group were significantly lower than the control group (*P* < 0.05), as shown in Table 3.

### 3.3. Comparison of T Cell Subset Levels before and after Treatment in the Two Groups of Patients

T lymphocyte subsets mediate cellular immunity, have antiviral and immune regulation functions, and their functions mainly depend on the relative composition of CD4+ and CD8+. Before treatment, there was no statistical difference in CD4+, CD8+, and CD4+/CD8+ between the two groups, and they were comparable. Within group comparison, the levels of CD4+ and CD4+/CD8+ in the two groups were increased, and the level of CD8+ was decreased (*P* < 0.05). CD4+ and CD4+/CD8+ in the observation group were higher and CD8+ was lower than the control group (*P* < 0.05), as shown in Figure 1.

### 3.4. Comparison of the Levels of Inflammatory Factors in the Two Groups before and after Treatment

There were no significant differences in serum inflammatory factors between the two groups before treatment. After 1 week of treatment, the level of IL-6 in the observation group was significantly lower than that in the control group, *P* < 0.05. There were no significant differences in other inflammatory factors between the two groups. After 2 weeks of treatment, the levels of IL-6, TNF-ɑ, IFN-*γ*, and CRP in the observation group were lower than those in the control group, *P* < 0.05. There was no statistically significant difference in WBC levels between the two groups, as shown in Table 4.

### 3.5. Adverse Drug Reactions in the Two Groups

The adverse reactions of the two groups of children during the treatment process were recorded in detail. The final statistics showed that the main adverse reactions were vomiting, diarrhea, and mild rash, and they were all mild and did not affect the treatment. During the treatment period, 2 cases of vomiting, 1 case of diarrhea, and 1 case of mild rash occurred in the control group, and no other obvious adverse reactions were found, and the incidence of adverse reactions was 11.76%. There was 1 case of vomiting and 1 case of diarrhea in the observation group, and no other obvious adverse reactions were found, and the incidence of adverse reactions was 5.88%. There was no significant difference in the incidence of adverse reactions between the two groups (*P* > 0.05) (Table 5).

## 4. Discussion

*Mycoplasma pneumoniae* pneumonia (MPP) is the more common pneumonia in childhood. In recent years, its incidence has been increased year by year, accounting for about 15% to 20% of paediatric pneumonia. *Mycoplasma pneumoniae* is the pathogen of MPP, and its pathogenesis is that *Mycoplasma pneumoniae* directly induces respiratory diseases by invading the respiratory tract. In addition to invading bronchopulmonary tissue, MPP can also cause diseases other than the respiratory system. Therefore, active and effective treatment of children with MPP is extremely important.

Pneumonia asthma is the most common type of pulmonary disease in pediatrics. Western medicine calls pneumonia asthma as bronchopneumonia, while traditional Chinese medicine belongs to the category of “pneumonia asthma.” Western medicine treatment mostly uses sensitive antibiotics macrolides, but the drug resistance is high and the curative effect is not good. In recent years, the clinical research on the infection of *Mycoplasma pneumoniae* in children has gradually deepened, and the traditional Chinese medicine syndrome differentiation and treatment plan is used to treat this disease, and the effect is more prominent. To analyze the treatment mechanism of traditional Chinese medicine, that is, to regulate the deficiency and excess of cold and heat in the body, promote the elimination of phlegm and phlegm in the lungs, and then smooth the qi stagnation and blood stasis, improve immunity, and finally play the role of strengthening the body and eliminating pathogens. In the clinical treatment of Chinese medicine, the most commonly used prescriptions are to resolve phlegm and relieve cough and to clear heat and detoxify.

The pathogenesis of mycoplasma pneumonia is related to *Mycoplasma pneumoniae* invasion and immune dysfunction. During the infection of mycoplasma pneumonia, a large amount of inflammatory responses will be produced, and the overexpression of inflammation can promote the occurrence and development of mycoplasma pneumonia and aggravate the disease [14,15]. CRP, IL-6, and TNF-*α* are the most important cells mediating early inflammatory response, and their levels can accurately reflect the degree of mycoplasma pneumonia infection and the outcome of disease [16–19]. Th1/Th2 immune response plays an important role in the pathogenesis of MPP. Among them, IL-6 is mainly an inflammatory factor mediated by Th2 cells, which plays a central role in acute inflammatory response. Overexpression of IL-6 often leads to persistent inflammation and even irreversible lung tissue damage [20,21]. IFN-*γ* is mainly produced by Thl cells, which can activate monocytes and macrophages. On the one hand, IFN-*γ* can assist in the differentiation of T lymphocytes, thereby enhancing cellular immune function. On the other hand, IFN-*γ* can cause the overexpression of respiratory endothelial cell adhesion factors, cause the proliferation and chemotaxis of inflammatory cells, release a large number of inflammatory mediators, and aggravate airway damage. Modern pharmacological studies have found that honeysuckle in Jiedu Pingsou Decoction can promote the phagocytosis of white blood cells and inflammatory cells. The active ingredient artemisinone can directly kill and inhibit influenza virus, inhibit pathogenic bacteria, and effectively inhibit the production of endogenous pyrogen and inflammatory factor IFN-*γ*.

In this study, the observation group used Jiedu Pingsou Decoction and azithromycin for the comprehensive treatment of children with mycoplasma pneumonia. The results of the study showed that compared with the control group with azithromycin alone, after treatment, the total effective rate was 94.12% in the observation group and 82.35% in the control group. The curative effect of the observation group was better than that in the control group, and the incidence of adverse reactions in the observation group was significantly lower than that in the control group (*P* < 0.05). The disappearance time of lung rales, cough, fever, and wheezing was significantly shorter than that of the control group (*P* < 0.05). The levels of CD8+, CRP, TNF-*α*, IFN-*γ*, IL-6, and IL-10 were lower than those before treatment, and the improvement in the observation group was better than that in the control group (*P* < 0.05). The levels of CD3+, CD4+, and CD4+/CD8+ were higher than those before treatment, and the improvement in the observation group was better than that in the control group (*P* < 0.05). The results of the study showed that the expression levels of CRP, IL-6, and TNF-*α* in the combined treatment were significantly lower than those in the single treatment with Western medicine, indicating that the combined treatment could reduce the level of inflammation and promote disease outcome. However, due to the limited number of patients participating in the study, the data have limitations.

In conclusion, Jiedu Pingsou Decoction combined with azithromycin can effectively improve the symptoms and signs of MPP and reduce the overexpression of inflammatory factors such as IFN-*γ*, TNF-*α*, and IL6. Jiedu Pingsou Decoction combined with azithromycin can quickly and effectively improve the clinical symptoms of children and reduce the incidence of adverse reactions. Jiedu Pingsou Decoction combined with azithromycin is more effective than pure azithromycin, which is safe and effective and is worthy of clinical application.

## Figures and Tables

**Figure 1:** Comparison of T cell subset levels before and after treatment in children with mycoplasma pneumonia in two groups.

**Table 1:** Comparison of general data of two groups of children.

Groups	Control group	Observation group	*χ* ^2^/P
*Gender*			0.06
Male	21	20	
Female	13	14	
Age	7.32 ± 2.13	7.29 ± 2.10	0.95
Course of disease	6.26 ± 1.21	6.24 ± 1.23	0.92

**Table 2:** Comparison of clinical efficacy between the two groups of patients.

Group	Significantly effective	Effective	Ineffective	Effective efficiency (%)
Control group	14	14	6	82.35
Observation group	17	15	2	94.12

**Table 3:** Comparison of clinical symptom scores between the two groups before and after treatment.

Group	Cough		Fever		Pulmonary rales	
	Before treatment	After treatment	Before treatment	After treatment	Before treatment	After treatment
Observation group	2.06 ± 0.72	0.62 ± 0.11	1.89 ± 0.77	0.43 ± 0.15	1.89 ± 0.63	0.67 ± 0.24
Control group	1.98 ± 0.75	1.25 ± 0.35	2.16 ± 0.81	1.22 ± 0.49	2.05 ± 0.82	1.51 ± 0.67
T	0.44	10.02	1.41	9.09	0.91	9.42
P	0.66	<0.001	0.16	<0.001	0.37	<0.001

**Table 4:** Comparison of the levels of inflammatory factors in the two groups of patients.

Groups	Times	WBC (×109 L^−1^)	IL-6/(ng·mL^−1^)	IL-10/(ng·mL^−1^)	IFN-*γ*/(ng·mL^−1^)	TNF-ɑ/(ng·mL^−1^)	CRP (ng·mL^−1^)
Control group	On admission	9.03 ± 2.81	20.68 ± 4.31	36.75 ± 6.85	26.87 ± 4.73	2.72 ± 0.53	13.42 ± 2.96
	1 week later	9.08 ± 2.83	17.98 ± 5.03	29.35 ± 4.23	21.75 ± 4.52	2.15 ± 0.42	11.23 ± 2.46
	2 weeks later	8.98 ± 2.75	14.02 ± 5.22	21.84 ± 4.32	15.45 ± 3.85	1.44 ± 0.31	8.63 ± 1.85

Observation group	On admission	8.90 ± 2.65	22.87 ± 4.87	38.01 ± 6.52	27.17 ± 4.85	2.91 ± 0.55	13.73 ± 3.03
	1 week later	8.65 ± 2.58	15.57 ± 3.99	22.06 ± 3.53	18.64 ± 4.03	1.83 ± 0.40	9.04 ± 1.31
	2 weeks later	8.74 ± 2.63	11.06 ± 3.01	15.61 ± 3.21	11.13 ± 3.42	0.87 ± 0.14	3.41 ± 0.74

**Table 5:** Comparison of the incidence of adverse reactions.

Groups	Vomit	Diarrhea	Mild rash	Adverse reaction rate (%)
Control group	2	1	1	11.76
Observation group	1	1	0	5.88

## Data Availability

The data that support the findings of this study are available on reasonable request from the corresponding author.
